The article "miR-302a-3p Promotes Radiotherapy Sensitivity of Hepatocellular Carcinoma by Regulating Cell Cycle via MCL1" was published in 2022. Journal: Comput Math Methods Med.

# miR-302a-3p Promotes Radiotherapy Sensitivity of Hepatocellular Carcinoma by Regulating Cell Cycle via MCL1

**DOI:** 10.1155/2022/1450098

**Published:** 2022-10-10

**Authors:** Zifeng Yang, Menglong Zhang, Jian Zhang, Cunkun Chu, Bijuan Hu, Liyin Huang

**Affiliations:** ^1^Department of Interventional Radiology, The Fifth People's Hospital of Jinan, Jinan, 250000 Shandong, China; ^2^Department of Minimally Invasive Intervention, Ganzhou People's Hospital, Ganzhou, Jiangxi 341000, China; ^3^Department of Pathology, Ganzhou People's Hospital, Ganzhou, Jiangxi 341000, China; ^4^Shandong First Medical University & Shandong Academy of Medical Sciences, Jinan, Shandong 250000, China; ^5^Department of Ultrasonography, Ganzhou People's Hospital, Ganzhou, Jiangxi 341000, China

## Abstract

**Background:**

The relationship between tumor suppressor gene miR-302a-3p and radiotherapy for hepatocellular carcinoma (HCC) remains unclear. This study intended to illustrate the molecular mechanism how miR-302a-3p regulated radiotherapy sensitivity of HCC.

**Methods:**

miR-302a-3p expression in HCC tissues and cells was examined by qRT-PCR. The effect of miR-302a-3p on HCC radiotherapy sensitivity were detected by CCK-8, colony formation, and flow cytometry assays. The expression levels of cell cycle-related proteins were detected by Western blot. The influence of miR-302a-3p on radiotherapy sensitivity of HCC was further investigated via cell cycle inhibitor (Caudatin) treatment. The target gene (MCL1) of miR-302a-3p was obtained by bioinformatics analysis, and their binding relationship was confirmed by RNA-binding protein immunoprecipitation assay. The mechanisms of miR-302a-3p regulating cell cycle and affecting radiotherapy sensitivity of HCC cells through MCL1 were further explored through the rescue experiments.

**Results:**

miR-302a-3p expression was remarkably reduced in radiotherapy-resistant tissues and cells of HCC. miR-302a-3p overexpression restored sensitivity of radiotherapy-resistant HCC cells to radiotherapy. Treatment with cell cycle inhibitor Caudatin could reverse suppressive effect of miR-302a-3p downregulation on sensitivity of HCC to radiotherapy. Additionally, miR-302a-3p could restrain MCL1 expression. *In vitro* cell assays further revealed that miR-302a-3p/MCL1 axis could enhance radiotherapy sensitivity of HCC cells by inducing G0/G1 arrest.

**Conclusions:**

miR-302a-3p facilitated radiotherapy sensitivity of HCC cells by regulating cell cycle via MCL1, which provided a new underlying target for radiotherapy resistance of HCC patients.

## 1. Introduction

Hepatocellular carcinoma (HCC) ranks fifth in prevalence of all cancers and second in cancer-related deaths worldwide [1]. The prognosis of HCC was poor with a 5-year survival rate of less than 30% [2]. However, due to unapparent symptoms at the early stage, most HCC patients are detected at an advanced stage, at which time patients cannot tolerate a surgical resection [3]. Radiation therapy is especially important for patients who are not eligible for a resection. The mainstream radiotherapy currently is the radiation therapy with a particle accelerator [4]. In addition, recent studies have shown that radioactive iodine-125 particle implantation therapy is an effective nonsurgical treatment for HCC patients who are unable to undergo resection. Iodine-125 particles are synthetic radionuclides that emit X- and *γ*-rays, which can damage tumor DNA and thus cause free radical production in tissues, which in turn kill tumor cells [5]. Currently, the feasible and well-tolerated radiotherapy has gradually become a noninvasive treatment for local ablation of HCC patients. However, radiotherapy-induced radiation resistance has seriously affected the control effect of radiotherapy on tumor [6]. The generation of radiotherapy resistance is related to many biological factors; the specific mechanism remains unclear. Therefore, elucidating the molecular mechanisms involved in radiotherapy resistance may help to explore therapeutic targets to improve the effectiveness of radiotherapy, thus achieving better therapeutic outcomes in HCC patients.

The article "miR-302a-3p Promotes Radiotherapy Sensitivity of Hepatocellular Carcinoma by Regulating Cell Cycle via MCL1" was published in 2022. Journal: Comput Math Methods Med.

MicroRNAs (miRNAs) play imperative regulatory roles in multiple biological and pathological processes of cancer [7]. Accumulating evidence has found that miRNAs affect radiotherapy resistance of various types of malignant tumors. For example, miR-612 was bound by TRPM2-AS in gastric cancer to increase FOXM1 expression and enhance radiotherapy resistance of gastric cancer [8]. MiR-208a could promote proliferation and radiotherapy resistance of lung cancer cells through targeting p21 [9]. In addition, miR-302a-3p can be a tumor suppressor in endometrial cancer, non-small-cell lung cancer, and melanoma [10–12], suggesting a tight relationship between miR-302a-3p and antitumor radiotherapy resistance. However, no studies have been reported on regulation of radiotherapy resistance of HCC via miR-302a-3p. Therefore, the present study preliminarily explored the potential impact and mechanism of miR-302a-3p on HCC radiotherapy resistance.

DNA damage response induced by ionizing radiation is a highly complex and coordinated system. Ionizing radiation can affect cell cycle progression by activating DNA damage checkpoints, which are specific points that prevent or slow down the cell from entering the next stage in the cell cycle [13]. The G2/M checkpoint is modulated by many proteins in eukaryotic cells, like cell division cycle 2 protein (Cdc2) and cyclin B protein (cyclin B), and reduced expression of Cdc2 and cyclin B can trigger G2/M arrest [14]. It is noteworthy that the radiosensitivity of cells shows varying characteristics in different cell cycle phases [15]. Specifically, G2/M phase is the most sensitive stage to radiation, while cells in S phase are the most resistant to radiation. Therefore, drugs that alter the course of the cell cycle are usually effective radiotherapy modulators [16, 17]. In addition, cyclin-dependent kinases (CDKs) have been shown to drive normal cells from G1 phase into the cell cycle process. Storch and Cordes [18], for example, found that CDK9 loss delayed cell transition from G1 to S phase, thereby enhancing radiotherapy sensitivity of head and neck squamous cell carcinoma cells. It seems that cell cycle condition correlates much to the efficacy of radiotherapy. Therefore, we assumed that miR-302a-3p enhances radiotherapy sensitivity by modulating cell cycle in HCC.

The article "miR-302a-3p Promotes Radiotherapy Sensitivity of Hepatocellular Carcinoma by Regulating Cell Cycle via MCL1" was published in 2022. Journal: Comput Math Methods Med.

Herein, we revealed that miR-302a-3p expression is related to tumor radiotherapy resistance, and further cell experiments found that miR-302a-3p could induce G0/G1 arrest and enhance the radiotherapy sensitivity of HCC. Our study experimentally proved that miR-302a-3p regulated cell cycle progression and facilitated radiotherapy sensitivity of HCC by downregulating MCL1 expression. These findings shed new insights into the mechanism of radiotherapy resistance of HCC and provided theoretical basis for miR-302a-3p as a promising radiotherapy sensitization target.

## 2. Materials and Methods

### 2.1. Bioinformatics Analysis

The mRNA expression profile of HCC was obtained from TCGA database, and then, the TargetScan (http://www.targetscan.org/vert_72/), miRDB (http://mirdb.org/), and starBase (http://starbase.sysu.edu.cn/) databases were used to predict downstream target genes of miR-302a-3p to obtain the differentially expressed mRNAs with binding site to miR-302a-3p. The predicted results were intersected with differentially downregulated mRNAs. Finally, the target gene was determined through correlation analysis.

### 2.2. Patient Tissues

With the approval of the Ethics Committee of Ganzhou People's Hospital, we collected 30 HCC tissue samples from patients who were sensitive or resistant to radiotherapy. The mean age of the patients included in this study was 60.26 years, including 13 females and 17 males. All the patients were in intermediate and advanced clinical stages. Cancer tissue sample collection was performed after the patients received the first radiotherapy. All samples were from patients receiving radical radiotherapy without a distant metastasis in Ganzhou People's Hospital. Samples were taken during surgery and then quickly frozen and stored at -80°C. Radiotherapy was performed according to standard treatment regimens, and efficacy was assessed at the end of radiotherapy to determine whether patients (and corresponding specimens) are resistant or sensitive to radiotherapy. All patients had signed the informed consents.

The article "miR-302a-3p Promotes Radiotherapy Sensitivity of Hepatocellular Carcinoma by Regulating Cell Cycle via MCL1" was published in 2022. Journal: Comput Math Methods Med.

### 2.3. Cell Culture and Radiation Treatment

Human HCC cell line HepG2 (BNCC338070) was provided by BeNa Culture Collection (BNCC, China). HepG2 cells were cultured in DMEM +10% fetal bovine serum (FBS) medium and placed in an incubator at 37°C with 5% CO_2_. The establishment of radiation-resistant HCC cells was performed as per the method described by Chen et al. [19]. Specifically, the HepG2 cells were treated with 6-MV X-rays generated by a linear accelerator (Varian 2300EX, dose rate of 2 Gy/min; Varian, USA). The cells were cultured after the initial radiation of 2 Gy and subcultured twice. The surviving cells were then exposed to a series of gradually increasing radiation doses (4, 6, 8, and 10 Gy) twice. The total radiation dose was 50 Gy, and the whole selection process was finished within 6 months. The final surviving cells were defined as HepG2/RR (radiation-resistant). We used parental HepG2 cells as controls and were defined as HepG2/RS (radiation-sensitive). HepG2/RR and HepG2/RS were cultured at 37°C for 24 h before further analyses.

### 2.4. Cell Transfection

miR-302a-3p mimic (miR-mimic), miR-302a-3p inhibitor (miR-inhibitor), and their negative controls (mimic-NC or NC-inhibitor) were all provided by Ribobio (China). The plasmids of miR-mimic/miR-NC, miR-inhibitor/NC-inhibitor, and oe-NC/oe-MCL1 were transfected into HCC cell line HepG2/RR by using Lipofectamine 2000 kit (Invitrogen, USA). The cells were then treated with X-rays and cultured for 24 h for following experiments.

### 2.5. Cell Cycle Inhibitors Treat Cells

Caudatin (Medherb Biotechnology, China) was dissolved in dimethyl sulfoxide, and HepG2/RR cells were treated with 100 *μ*M Caudatin for 24 h for subsequent experiments.

### 2.6. qRT-PCR

Total RNA was separated with RNAiso Plus (Takara, Japan), and Prime Script TM RT Master Mix (Takara, Japan) was recommended for reverse transcription. qPCR was completed on SYBR Premix Ex Taq II (Takara, Japan). The operation for RNA extraction and PCR analysis were carried out as per the methods described by predecessors [20]. U6 snRNA and GAPDH were served as internal references to quantify miRNA and mRNA in cells. qPCR was performed with StepOnePlus Real-Time PCR system (AB, USA). The PCR results were quantified by 2^−ΔΔCt^, and the experiment was repeated 3 times.  Table 1 exhibits the primer sequences.

The article "miR-302a-3p Promotes Radiotherapy Sensitivity of Hepatocellular Carcinoma by Regulating Cell Cycle via MCL1" was published in 2022. Journal: Comput Math Methods Med.

### 2.7. Western Blot

The required proteins were extracted from cells, and the protein concentration was determined by BCA kit (Beyotime, China). The same amount of proteins (50 *μ*g) was added to each well of SDS-PAGE gel. After electrophoresis for 1.5 h, the protein was transferred to PVDF membrane. The PVDF membrane was placed in 0.5% skim milk powder and blocked at room temperature for 1.5 h. The PVDF membrane was then probed with the primary antibodies and incubated overnight (4°C). After washing three times with TBST, the membrane was placed in the second antibody and incubated for 2 h (room temperature). ECL kit (Thermo Scientific, USA) was used for color developing. Detailed steps of Western blot were performed according to previously described methods [21], and the experiment was repeated 3 times. The primary antibodies included rabbit anti-cyclin D1 (ab134175), rabbit anti-cyclin E1 (ab224819), rabbit anti-P27 (ab137736), and rabbit anti-GAPDH (ab181602), and the secondary antibody was goat anti-rabbit IgG (ab205718), all purchased from Abcam (Abcam, UK).

### 2.8. CCK-8 Assay

To investigate sensitivity of HepG2/RS and HepG2/RR cells to radiotherapy, cells that had received different ionizing radiation doses (0, 2, 4, 6, 8, and 10 Gy) were inoculated into a 96-well plate (2 × 10^4^ cells/well). After 24 h of culture, CCK-8 reagent was added as per the instructions of CCK-8 kit (Beyotime, China), and absorbance of cells was determined at 450 nm.

To detect sensitivity of miR-302a-3p-transfected HepG2/RR cells to radiotherapy, cell viability was detected on d1, d2, d3, d4, d5, d6, d7, and d8 according to kit instructions after 8 Gy radiation treatment, and the experiment was repeated 3 times.

### 2.9. Colony Formation Assay

Transfected or untransfected HepG2/RR cells were plated into a 6-well plate (1 × 10^3^ cells per well). The cells received different ionizing radiation doses (0, 2, 4, 6, 8, and 10 Gy). Culture medium was replaced after 24 h, and then, the cells were maintained for 10-14 days. When visible cell colonies appeared, the medium was discarded. The cells were rinsed 3 times with cold PBS, followed by fixing with paraformaldehyde for 15 min and staining with 0.5% crystal violet solution for 15 min. After washing with PBS, cells were dried, and colonies were photographed and counted using camera.

### 2.10. Flow Cytometry

For cell cycle detection, transfected cells in each group were cultured to logarithmic growth phase. After receiving 8 Gy ionizing radiation and being cultured for 24 h, the cells were digested with trypsin, washed with PBS, and fixed in 70% ethanol overnight. Then, the cells were dyed with propidium iodide. The distribution of cell cycle was analyzed by flow cytometry.

The article "miR-302a-3p Promotes Radiotherapy Sensitivity of Hepatocellular Carcinoma by Regulating Cell Cycle via MCL1" was published in 2022. Journal: Comput Math Methods Med.

### 2.11. RIP Assay

RIP assay was carried out according to the steps of Zhang et al. [22]. In brief, HepG2 cells were treated with miR-NC or miR-mimic. 48 h later, the transfected cells were subjected to RIP assay with the Magna RIP™ RNA Binding Protein Immunoprecipitation Kit (Millipore, USA). Subsequently, the cells were probed with anti-Ago2 antibody or negative control IgG. The relative enrichment degree of MCL1 was determined by qRT-PCR.

### 2.12. Data Analysis

Data graphs and data analysis in this paper were plotted and analyzed using GraphPad Prism 8 (GraphPad Software, USA), and intergroup comparison was performed using ANOVA or *t-*test. The data were presented as the mean ± standard deviation (SD) from at least three independent experiments. *p* < 0.05 meant that the difference was significant.

## 3. Results

### 3.1. miR-302a-3p Was Lowly Expressed in Radiotherapy-Resistant HCC Tissues and Cells

To study the role of miR-302a-3p in regulating HCC resistance to radiotherapy, we first measured the expression of miR-302a-3p expression in tumor tissues of HCC patients with radiotherapy sensitivity or radiotherapy resistance. The result displayed that miR-302a-3p was dramatically underexpressed in tumor tissues with radiotherapy resistance (Figure 1(a)). Then, HepG2 cells were used to establish radiotherapy-sensitive HepG2/RS and radiotherapy-resistant HepG2/RR. qRT-PCR was utilized to detect miR-302a-3p level in HepG2/RS and HepG2/RR cells. The result displayed a notable reduction in miR-302a-3p expression in radiotherapy-resistant HepG2/RR cells compared to its parental radiotherapy-sensitive HepG2/RS cells (Figure 1(b)). Subsequent CCK-8 result displayed that radiotherapy resistance of HepG2/RR cells was significantly enhanced compared with HepG2/RS, indicating that HepG2/RR cells obtained higher radiotherapy resistance, with a median lethal radiation dose of 8 Gy (Figure 1(c)). In conclusion, we successfully constructed radiotherapy-sensitive HepG2/RS and radiotherapy-resistant HepG2/RR cells and found that miR-302a-3p was dramatically underexpressed in HCC tissues and cells with radiotherapy resistance.

### 3.2. miR-302a-3p Overexpression Enhanced Radiotherapy Sensitivity of HCC

To preliminarily explore effects of miR-302a-3p on cell viability, survival rate, and cycle of radiotherapy-resistant HCC cells, we constructed HepG2/RR cells with overexpression miR-302a-3p (miR-mimic) and its negative control (mimic-NC). First, the transfection efficiency of miR-302a-3p was evaluated by qRT-PCR, and the result indicated a prominent increase in miR-302a-3p expression in miR-mimic group (Figure 2(a)). Then, the cell viability was detected by CCK-8. It was demonstrated that miR-302a-3p overexpression remarkably reduced viability of HepG2/RR cells compared with control group (Figure 2(b)). Besides, the result of colony formation assay demonstrated that survival rate of HepG2/RR cells with miR-302a-3p mimic was notably reduced (Figure 2(c)) after cells were exposed to radiation, indicating that radiotherapy sensitivity of HepG2/RR cells was improved. Then, flow cytometry was adopted to detect cell cycle distribution in each treatment group. It was found that cells in G0/G1 phase were prominently increased and those in S phase were remarkably decreased in miR-mimic group (Figure 2(d)). Western blot analysis showed that expression levels of cyclin D1 and cyclin E1 were significantly downregulated, while expression of cell cycle regulator P27 was remarkably upregulated after miR-302a-3p overexpression (Figure 2(e)). In conclusion, these results indicated that overexpression of miR-302a-3p enhanced radiotherapy sensitivity, inhibited cell viability, and led to cell cycle arrest at G0/G1 phase.

The article "miR-302a-3p Promotes Radiotherapy Sensitivity of Hepatocellular Carcinoma by Regulating Cell Cycle via MCL1" was published in 2022. Journal: Comput Math Methods Med.

### 3.3. miR-302a-3p Enhanced Radiotherapy Sensitivity of HCC by Modulating Cell Cycle

To further analyze the impact of miR-302a-3p on sensitivity of HCC cells by affecting cell cycle, we set the following cell groups: negative control group (NC-inhibitor+DMSO), miR-302a-3p low expression group (miR-inhibitor+DMSO), and miR-302a-3p low expression with 100 *μ*M cell cycle inhibitor Caudatin group (miR-inhibitor+Caudatin). First, CCK-8 was utilized to detect effects of different treatments on cell viability. Compared to control group, the HepG2/RR cells with downregulated miR-302a-3p expression showed enhanced viability, which was reversed by the simultaneous addition of cell cycle inhibitor (Figure 3(a)). Then, colony formation assay was introduced to measure survival rate of HepG2/RR cells in each treatment group. The experimental result demonstrated that survival rate of HepG2/RR cells with downregulated miR-302a-3p was significantly increased after radiation exposure, while simultaneous addition of cell cycle inhibitor reversed effect of miR-302a-3p on survival rate of HepG2/RR cells (Figure 3(b)). Subsequently, flow cytometry was applied to analyze cell cycle distribution of each treatment group. According to the results, the number of G0/G1 phase cells was notably reduced in miR-inhibitor+DMSO group and prominently increased in miR-inhibitor+Caudatin group compared to NC-inhibitor+DMSO group (Figure 3(c)). Additionally, Western blot was applied to evaluate expression of cell cycle-related proteins. According to the experimental results, cyclin D1 and cyclin E1 expression was upregulated, and P27 expression was downregulated in miR-inhibitor+DMSO group compared to NC-inhibitor+DMSO group, while cyclin D1 and cyclin E1 expression was downregulated, and P27 expression was upregulated in miR-inhibitor+Caudatin group compared to miR-inhibitor+DMSO group (Figure 3(d)). These results implied that miR-302a-3p could make HCC cells sensitive to radiotherapy by regulating cell cycle.

The article "miR-302a-3p Promotes Radiotherapy Sensitivity of Hepatocellular Carcinoma by Regulating Cell Cycle via MCL1" was published in 2022. Journal: Comput Math Methods Med.

### 3.4. miR-302a-3p Enhanced Radiotherapy Sensitivity of HCC Cells by Regulating Cell Cycle via MCL1

Studies have shown that miRNA mainly participates in the molecular regulatory pathway by regulating expression of target genes. We further explored downstream target mRNAs of miR-302a-3p through bioinformatics methods. First, differential analysis on the mRNAs in TCGA-HCC database were performed. Then, the obtained differentially downregulated mRNAs were intersected with the target genes of miR-302a-3p predicted by TargetScan, starBase, and miRDB databases. By this way, differential mRNAs with binding site to miR-302a-3p were obtained (Figure 4(a)). After reviewing the literature, we found that MCL1 was a key protein related to cell cycle [23] and that MCL1 was significantly overexpressed in tumor tissues with radiotherapy resistance (Figure 4(b)). Therefore, we selected MCL1 as the research object to explore its influence on the radiotherapy sensitivity of HCC cells. Subsequently, the binding site between miR-302a-3p and MCL1 was predicted by bioinformatics analysis (Figure 4(c)). The binding relationship between miR-302a-3p and MCL1 was further verified by RIP experiment, and the result showed that MCL1 was significantly enriched in miR-mimic cells (Figure 4(d)). To investigate whether miR-302a-3p can affect cell cycle progression by targeting MCL1, we first constructed miR-302a-3p overexpression cells (miR-mimic+oe-NC), MCL1 overexpression cells (mimic-NC+oe-MCL1), and miR-302a-3p and MCL1 simultaneous overexpression cells (miR-mimic+oe-MCL1) using HepG2/RR cells. According to qRT-PCR result, the mRNA expression of MCL1 was significantly reduced in miR-mimic+oe-NC group in comparison with control group, but it was recovered in miR-mimic+oe-MCL1 cotransfection group (Figure 4(e)). With regard to CCK-8 result, the viability of HepG2/RR cells in mimic-NC+oe-MCL1 group was enhanced compared to the mimic-NC+oe-NC, but it was restored in miR-mimic+oe-MCL1 group (Figure 4(f)). Then, flow cytometry result indicated the number of G0/G1 cells in mimic-NC+oe-MCL1 was significantly reduced compared to mimic-NC+oe-NC group, but the number in miR-mimic+oe-MCL1 group was recovered (Figure 4(g)). Western bolt was used to evaluate the expression of cell cycle-related proteins. According to the result, cyclin D1 and cyclin E1 expression was upregulated, and P27 expression was downregulated in mimic-NC+oe-MCL1 group compared to mimic-NC+oe-NC group, while expression levels of these proteins were recovered in miR-mimic+oe-MCL1 group (Figure 4(h)). These results indicated that miR-302a-3p could promote radiotherapy sensitivity of HCC cells by regulating HepG2/RR cell cycle progression via downregulation of MCL1.

The article "miR-302a-3p Promotes Radiotherapy Sensitivity of Hepatocellular Carcinoma by Regulating Cell Cycle via MCL1" was published in 2022. Journal: Comput Math Methods Med.

## 4. Discussion

Radiotherapy resistance is an important factor leading to clinical radiotherapy failure in HCC patients. Radiotherapy resistance can be attributed to the inherent radioresistance of tumor cells in hypoxic microenvironment or to the resistance acquired during hyperfraction radiotherapy [24]. Studies have shown that radiation exposure can increase the levels of intracellular free radical species, cause DNA strand breaks, and lead to subsequent dysfunction of some organelles such as mitochondria and endoplasmic reticulum [25]. These radiation-induced cellular events facilitate proapoptotic signal activation and ultimately cause tumor cell killing [26]. Nevertheless, the key molecules involved in radiation-induced radiotherapy resistance are still poorly understood. Hence, it is an urgent task to study the molecular mechanism of radiotherapy resistance and find new therapeutic targets, which are of great importance to overcome cancer radiotherapy resistance.

The regulatory mechanisms of miRNAs in the progression of many complex diseases have been extensively studied. miR-302a-3p plays a potential cancer-promoting role. For example, Zhang et al. [27] found that miR-302a-3p directly targets SOCS5 to promote STAT3 phosphorylation and induce transcription of STAT3 target genes, thereby promoting metastasis of pancreatic cancer cells. However, miR-302a-3p acts as an important tumor suppressor in most cases, where it inhibits the biological processes like proliferation, invasion, and migration of various human cancers, including HCC, colon cancer, and gastric cancer [28–30]. It is worth noting that miR-302a, as the precursor of miR-302a-3p, has been proved to participate in the inhibition of tumor chemotherapy resistance development [31, 32]. In addition, Liang et al. [33] discovered that miR-302a sensitizes radiation-resistant breast cancer cells to radiotherapy both *in vivo* and *in vitro*. Yu et al. [34] obtained similar results and found that miR-302a overexpression hampers proliferation of non-small-cell lung cancer, promotes cell apoptosis, and reduces cell radioresistance. Therefore, it is reasonable to speculate that miR-302a-3p is associated with HCC radiotherapy resistance. In this study, miR-302a-3p was remarkably downregulated in radiotherapy-resistant cells (HepG2/RR) compared with radiotherapy-sensitive cells (HepG2/RS). However, miR-302a-3p overexpression could enhance the radiotherapy sensitivity of HCC cells, confirming that miR-302a-3p mediated radiotherapy resistance in HCC.

The article "miR-302a-3p Promotes Radiotherapy Sensitivity of Hepatocellular Carcinoma by Regulating Cell Cycle via MCL1" was published in 2022. Journal: Comput Math Methods Med.

Radiation resistance is a complex cellular response involving many signaling pathways and genes. Ionizing radiation can induce DNA damage, including DNA single-strand break, DNA base damage, and DNA double-strand break [35]. In addition, DNA damage induced by ionizing radiation can activate a series of cell cycle checkpoints [36]. Hence, cell cycle checkpoint block is involved in the regulation of tumor radiotherapy resistance. For example, Wang et al. [37] showed that cyclin D1 and cyclin E1 are specific targets of miR-16-5p and that miR-16-5p overexpression can downregulate expression of cyclin D1 and cyclin E1 and induce cell cycle arrest in G0/G1 phase, which enhances radiosensitivity of prostate cancer cells. Although numerous studies have revealed the role of periodic checkpoint block in tumor radiotherapy resistance, there is little research on the regulatory role of miR-302a-3p. In the present study, *in vitro* cell experiments confirmed that miR-302a-3p induced cell arrest in G0/G1 phase by regulating expression of key cell cycle proteins cyclin D1, cyclin E1, and P27 and promoted the sensitivity of radiation-resistant HCC cells to radiotherapy, which was consistent with previous studies. In addition, this study predicted a new downstream target of miR-302a-3p, MCL1, through bioinformatics analysis, and verified the targeted relationship between the two. MCL1 has been proved to be overexpressed in many human cancers and contributes to cancer occurrence and inhibits apoptosis [38]. Specific targeting of MCL1 may overcome the antiapoptotic ability of malignant tumor cells. For example, BAG3 can upregulate MCL1 by downregulating miR-29b, thereby inducing chemotherapy resistance to paclitaxel in ovarian cancer [39]. In addition, Yu et al. found that MCL1 overexpression significantly inhibited mulanin-induced autophagy and cell cycle arrest in colorectal cancer cells [40]. In the present study, rescue experiments demonstrated that miR-302a-3p induced cell cycle arrest and promoted sensitivity of HCC cells to radiotherapy by targeting MCL1 expression, which was in accordance with the results of previous reports.

Our results confirmed that miR-302a-3p could enhance radiotherapy sensitivity of radiation-resistant HCC cells by regulating the cell cycle. In addition, our study revealed influences of miR-302a-3p/MCL1 axis on the radiotherapy sensitivity of HCC cells for the first time. However, the mechanism of miR-302a-3p enhancing the radiotherapy sensitivity of HCC was analyzed at the cellular level, which has not been verified *in vivo* at the animal level. Meanwhile, it also lacked the exploration of relevant signal pathways, which was the deficiency of this study. In summary, this study for the first time clarified the modulatory mechanism of miR-302a-3p in HCC radiotherapy resistance, suggesting that miR-302a-3p may be a potential sensitizer of radiotherapy. Our results provided new evidence for the radiotherapy resistance mechanism of HCC cells and can help overcome the difficulties in cancer radiotherapy in the future.

The article "miR-302a-3p Promotes Radiotherapy Sensitivity of Hepatocellular Carcinoma by Regulating Cell Cycle via MCL1" was published in 2022. Journal: Comput Math Methods Med.

## Figures and Tables

**Figure 1:** miR-302a-3p was underexpressed in radiotherapy-resistant HCC tissues and cells. (a) miR-302a-3p expression level in radiation-sensitive and radiation-resistant HCC tissues; (b) miR-302a-3p expression level in HepG2/SR and HepG2/RR cells; (c) cell viability of HepG2/RS and HepG2/RR cells under different radiation doses. ^∗^ represents *p* < 0.05.

**Figure 2:** miR-302a-3p overexpression enhanced the radiotherapy sensitivity of HCC cells. (a) miR-302a-3p expression in HepG2/RR cells with miR-mimic/mimic-NC; (b) cell viability of HepG2/RR cells treated for different days with 8 Gy radiation dose; (c) survival rate of HepG2/RR cells treated with different radiation doses; (d) cell cycle distribution of HepG2/RR cells treated with 8 Gy radiation doses; (e) expression of cyclins in HepG2/RR cells. ^∗^ represents *p* < 0.05.

**Figure 3:** miR-302a-3p enhanced radiotherapy sensitivity of HCC cells by regulating cell cycle. (a) Cell viability of HepG2/RR cells treated for different days with 8 Gy radiation dose; (b) survival rate of HepG2/RR cells treated with different radiation doses; (c) cell cycle phase distribution of HepG2/RR cells treated with 8 Gy radiation doses; (d) expression of cyclins in HepG2/RR cells. ^∗^ represents *p* < 0.05.

**Figure 4:** miR-302a-3p enhanced radiotherapy sensitivity of HCC cells by regulating cell cycle via MCL1. (a) Venn diagram of predicted mRNAs of miR-302a-3p and downregulated differential mRNAs; (b) MCL1 expression in radiation-sensitive and radiation-resistant tissues of HCC patients; (c) schematic diagram of the binding between MCL1 and miR-302a-3p sequences predicted by starBase; (d) binding relationship between miR-302a-3p and MCL1 verified by RIP experiment; (e) MCL1 mRNA expression of HepG2/RR cells in different treatment groups; (f) cell viability of HepG2/RR cells treated for different days with 8 Gy radiation dose; (g) cell cycle distribution of HepG2/R cells treated with 8 Gy radiation dose; (h) the expression of cyclins in HepG2/RR cells. ^∗^*p* < 0.05 vs. (mimic-NC + oe-NC), ^#^*p* < 0.05 vs. (mimic-NC+oe-MCL1).

The article "miR-302a-3p Promotes Radiotherapy Sensitivity of Hepatocellular Carcinoma by Regulating Cell Cycle via MCL1" was published in 2022. Journal: Comput Math Methods Med.

**Table 1:** Primer sequence for qRT-PCR analysis.

Gene	Sequence	
miR-302a-3p	Forward primer	5′-ACACUCCAGCUGGGAGUGGUUUUGUACCUUC-3′
	Reverse primer	5′-CUCAACUGGUGUCGUGGAGUCGGCAAUUCAGUUGAGUCGUGAAU-3′

U6	Forward primer	5′-CTCGCTTCGGCAGCAC-3′
	Reverse primer	5′-AACGCTTCACGAATTTGCGT-3′

MCL1	Reverse primer	5′-GGGCAGGATTGTGACTCTCATT-3′
	Forward primer	5′-GATGCAGCTTTCTTGGTTTATGG-3′

GAPDH	Reverse primer	5′-AAGGTGAAGGTCGGAGTCAA-3′
	Forward primer	5′-AATGAAGGGGTCATTGATGG-3′

## Data Availability

The data that support the findings of this study are available on request from the corresponding author.
